# Comparison of Contrast-Enhanced Spectral Mammography and Contrast-Enhanced MRI in Screening Multifocal and Multicentric Lesions in Breast Cancer Patients

**DOI:** 10.1155/2022/4224701

**Published:** 2022-04-06

**Authors:** Lei Feng, Lei Sheng, Litao Zhang, Na Li, Yuanzhong Xie

**Affiliations:** ^1^Department of Radiology, Jining No. 1 People's Hospital, Jining 272013, China; ^2^Department of Clinic Imaging, Taian City Central Hospital, Affiliated Hospital of Qingdao University, Taian 271000, China; ^3^Graduate School, Shandong First Medical University and Shandong Academy of Medical Sciences, Taian 271000, China

## Abstract

**Objectives:**

We aimed to determine the difference between contrast-enhanced spectral mammography (CESM) and contrast-enhanced magnetic resonance imaging (CE-MRI) in detecting multifocal and multicentric breast cancer (MMBC).

**Methods:**

: This study was conducted among breast cancer patients between July 1, 2017, and May 30, 2021. The sensitivity, specificity, and accuracy of CESM and CE-MRI in the diagnosis of MMBC were evaluated with pathological results as the gold standard.

**Results:**

A total of 188 lesions were detected in 54 patients with MMBC, including 177 breast cancer and 11 benign lesions. Based on CESM and CE-MRI, 4 false-positive cases and 3 false-negative cases and 7 false-positive cases and 1 false-negative case, respectively, were found. The accuracy of CESM was higher than that of MRI (96.3% vs 95.7%), and the specificity was higher than that of MRI (63.6% vs 36.4%). There were no significant differences in the sensitivity, specificity, and accuracy for the detection of MMBC between CESM and CE-MRI (*p* = 0.500; *p* = 0.250; *p* = 0.792).

**Conclusion:**

CESM is an effective method for the detection of MMBC, which is consistent with the sensitivity and accuracy of CE-MRI.

## 1. Introduction

Breast cancer is one of the most common fatal malignancies in women. Preoperative assessment when choosing between total and conservative mastectomy depends on the extent of the cancer and whether the cancer is multifocal or multicentric [1, 2]. Compared with breast cancer patients presenting with a single focal lesion, multifocal and multicentric breast cancer (MMBC) showed a higher risk of lymph node metastasis and aggression, a higher degree of malignancy, as well as a poorer prognosis [3, 4]. The incidence of MMBC has a wide variation (6%–60%) among different clinical studies, mostly due to the lack of a standardized classification [5]. Therefore, a comprehensive preoperative imaging evaluation, such as first-line imaging evaluation by mammography and ultrasonography (US) followed by contrast-enhanced magnetic resonance imaging (CE-MRI), is essential for patients suspected with multiple breast cancers.

Mammography is a conventional modality of breast screening or clinical diagnosis of breast cancers. The cancer detection sensitivity is only about 50% to 60% in dense breasts because of poor contrast between the cancer and the background [6]. Thus, there is a high possibility of underdetection. US is commonly used for cancer detection, as well as preoperative evaluation of cancer status due to the advantages of being handheld, convenient, and radiation-free, but single US application usually showed poor consistency with pathological diagnosis [7]. A few studies have proposed the limitations of classic ultrasonographic differentiation between benign and malignant masses. Ultrasonography-based texture analysis (USTA) offers a new perspective. It is unclear whether the parameters can reflect the histopathological characteristics of lesions [8]. Recently, preoperative contrast-enhanced ultrasonography only showed good predictive value for the sentinel lymph node detection in patients with breast cancer [8]. CE-MRI is considered to be one of the most accurate imaging methods for the diagnosis of breast cancer [9]. Although it has a high sensitivity for identifying MMBC from 88% to 100%, the specificity and positive predictive value (PPV) of CE-MRI are limited as both benign and malignant lesions presenting enhancement [10]. Additionally, it is more expensive, time-consuming, and not easily accessible compared with mammography.

Recently, an emerging imaging technique of contrast-enhanced spectral mammography (CESM) provides a low-energy mammogram (LE-MG) and a recombined subtracted mammogram (RSM) after intravenously administering iodinated contrast medium images in the same session of examination within a short time. CESM allows both a morphologic evaluation comparable to routine digital mammography and a simultaneous assessment of tumor neovascularity as an indicator of malignancy [11].

Preliminary studies indicated that CESM showed an extremely high sensitivity to breast cancer. To date, a few studies have focused on the comparison of the screening efficiency for malignancies between CESM and CE-MRI [12, 13]. The studies reported better accuracy and specificity and a decreased false-positive rate of CESM in breast cancer detection than those of MRI. Recently, a few studies have been available to assess the effectiveness of the radiomics analysis of CESM in discriminating between breast cancers and background parenchymal enhancement (BPE), as well as to discrimination of benign and malignant breast lesions [14, 15]. However, to the best of our knowledge, few studies have focused on the diagnostic performance of CESM in the diagnosis of MMBC [1]. Accordingly, this study aimed to compare the diagnostic performance of CESM in the discovery of MMBC compared with CE-MRI to determine whether CESM could result in changes to surgical management.

## 2. Materials and Methods

### 2.1. Inclusion and Exclusion Criteria

Between July 1, 2017, and May 30, 2021, MMBC patients were included in this study based on the following criteria: (1) the final diagnosis with MMBC was established via core needle biopsy under the guidance of US and/or surgery. Histopathologic diagnosis was utilized as the standard; (2) MRI and CESM were scheduled within 3 days in premenopausal women and within 14 days in postmenopausal women; and (3) we included all types of breast (A–D) based on the American College of Radiology (ACR). Patients were excluded based on the following criteria: (1) the patient with single focal breast cancer; (2) the patient was pregnant or lactating; (3) the patient with claustrophobia; (4) the patient received implanted pacemakers or metal implants previously; and (5) the patient with hyperthyroidism, or a history of allergy to iodine or gadolinium contrast agent, or severe hepatorenal dysfunction with a glomerular filtration rate of <30 ml/min.

### 2.2. CE-MRI Examinations

The 3.0 T superconducting MR instrument (Magnetom Aera; Siemens, Erlangen, Germany) equipped with the 16-channel breast coil was used for the CE-MRI scan. The patients were in a prone position with bilateral breasts loosing naturally within the breast-dedicated coils. After conventional plain scan, diffusion weighted imaging (DWI) was performed, followed by CE-MRI scan. The contrast medium (Gd-DTPA) was used and injected at a dose of 0.2 mmol/kg and a rate of 2 ml/s. The conventional plain scan sequences were as follows: T1WI sequence (TR 6.0 ms, TE 2.46 ms), fast reversal recovery of T1WI sequence by fat suppression (TR 4,000 ms, TE 54 ms, slice thickness 4.0 mm), and bilateral mammary sagittal T2WI sequence (TR 3,300 ms, TE 70 ms, slice thickness 4.0 mm); and horizontal axis DWI sequence: TR 4,730 ms, TE 47 ms, slice thickness 5.0 mm, *b* = 0, 400, 800 s/mm^2^. For the CE-MRI, fast 3D dynamic imaging fat suppression T1WI sequence was used: TR 4.66 ms, TE 1.70 ms, slice thickness 1.6 mm. One time phase was scanned before injection of Gd-DTPA, and six time phases were scanned again after injection with an interval of 64 sec. Then, the digital subtraction was performed on the transverse and coronal planes. For suspicious masses, a time-signal strength curve was added.

### 2.3. CESM Examinations

GE digital mammography equipment (Senographe Essential; GE Healthcare, Buc, France) was used for the CESM under the assistance of double-cylinder high-voltage syringe (Ulrich, Germany). Each patient received ioversol injection (1.5 ml/kg) via the radial vein, with a flow rate of 3 ml/s. About within 2 min after ioversol injection, the craniocaudal (CC) position of the affected breast was first photographed, and then the CC images of the healthy breast were obtained. The medial-lateral oblique (MLO) position of the affected breast was scanned, and then the MLO images of the healthy breast were obtained. The examination was completed within 6 min after injection. Briefly, a pair of LE-MG and high-energy MG is obtained, and then the images are subtracted from each other. After CESM, patients were recommended to drink more water, followed by observation for 30 min until presence of no adverse reactions.

### 2.4. Image Analysis

CESM and CE-MRI images were independently analyzed by three radiologists with 10-year working experience in breast cancer diagnosis who were blinded to patients' conditions. All the images were reviewed based on the criteria from the BI-RADS lexicon [16]. Digital mammography BI-RADS descriptors of lesions can be applied for the morphologic analysis of mass lesions on the low-energy MG imaging of CESM. The RSM of CESM images was evaluated using criteria related to contrast enhancement intensity and morphology according to the MRI part of the BI-RADS lexicon [17]. Subjective judgment of lesion enhancement was performed based on the scale of none, mild, moderate, and strong [18].

The lesions of a BI-RADS category of equal or less than 3 were diagnosed as benign, and those of above BI-RADS 4 (BI-RADS 4 A, B, C and BI-RADS 5) were diagnosed as malignant. For the detection of lesions, multifocal cancer was confirmed in the presence of two or more malignant focus in the same quadrant. Multicentric cancer was confirmed in cases of involvement of different quadrants.

### 2.5. Pathological Evaluation of Specimens

The specimens were fixed, embedded, and subjected to hematoxylin-eosin (HE) staining and immunohistochemical analysis. Pathological analysis was performed by pathologists with 10-year working experience based on the Pathological Classification and Diagnostic Criteria of Breast Tumors (2012) proposed by the World Health Organization (WHO) [19]. A caliper was utilized to assess the gross specimen for large specimens, while the small specimens were measured under a microscope.

### 2.6. Statistical Analysis

For statistical analysis, BI-RADS 1–3 and BI-RADS ≥ 4 were defined as suspicious benign and probably malignant, respectively. The chi-square test was used to compare the sensitivity, specificity, and accuracy in detecting MMBC between CESM and CE-MRI. With the pathological results as the criterion standard, the diagnostic accuracy was compared among different images. All statistical analysis was performed with IBM SPSS Statistics for Windows, version 20.0 (IBM Corp; Armonk, NY, USA) software. *p* < 0.05 was considered to be statistically significant.

## 3. Results

### 3.1. Patient Characteristics and Pathological Diagnosis

The study population consisted of 54 patients. All 54 patients were female (median age: 48.7 years; range: 33–73 years) and were proven to be MMBC (type A: 4; type B: 24; type C: 18; type D: 8) based on the guidelines proposed by the American College of Radiology (ACR). A total of 188 lesions were proven by pathology, including 11 benign lesions (5 lesions of fibroadenoma, 3 lesions of fibrocystic lesion with ductal hyperplasia, 2 lesions of breast adenosis with fibroadenoma, and 1 lesion of inflammation), and 177 lesions of malignant lesions. Of the 177 lesions, 69 lesions were invasive ductal carcinoma (IDC) including 9 lesions of invasive micropapillary carcinoma, and 1 lesion of mucinous carcinoma, together with 96 lesions of IDC with ductal carcinoma in situ (DCIS), 5 lesions of DCIS, 4 lesions of invasive lobular carcinoma, as well as 3 lesions of invasive lobular carcinoma with DCIS.

### 3.2. Comparison between the Efficiency of CESM and CE-MRI in the Diagnosis of MMBC

The results of TP, FP, FN, and TN by CESM and CE-MRI in detecting MMBC are shown in Table 1. The sensitivity, specificity, and accuracy rate of CESM in detecting MMBC were 98.3% (174/177), 63.6% (7/11), and 96.3% (181/188), respectively. For CE-MRI, the sensitivity, specificity, and accuracy rate were 99.4% (176/177), 36.4% (4/11), and 95.7% (180/188), respectively. There were no significant differences in the sensitivity, specificity, and accuracy between CESM and CE-MRI (*p* = 0.500; *p* = 0.250; *p* = 0.792, respectively) (Table 2, Figure 1).

Among the 177 malignant, 54 lesions showed clustered microcalcifications in the LE-MG imaging. 35 (64.8%, 35/54) lesions were assessed as BI-RADS 5. For CE-MRI, 22 (40.7%, 22/54) were diagnosed as BI-RADS 5 (Figure 2).

Among the 165 malignant lesions correctly detected by CESM, 160 (96.9%) lesions were IDC. Among the 160 IDC, there were 154 (96.3%) lesions with markedly heterogeneous enhancement similar to nipple enhancement. The other 6 lesions (3.7%) showed mild enhancement that were weaker than nipple enhancement (Figure 3).

## 4. Discussion

CE-MRI has been acknowledged as one of the most accurate imaging methods for the diagnosis of breast cancer [20]. In a previous study, Rabasco et al. reported a higher sensitivity (100%) and an accuracy rate (98.4%) of MRI in screening MMBC compared with mammography (40%, 92.5%), as well as the combination of mammography and US (57.1%, 92.5%) [21]. Our study demonstrated that CESM possessed a high sensitivity and might serve as a promising candidate for screening MMBC. There were no significant differences in the sensitivity, specificity, and accuracy between CESM and CE-MRI (*p* = 0.500; *p* = 0.250; *p* = 0.792, respectively).

CESM provided more comprehensive information for the diagnosis of MMBC. In the presence of the combination of LE-MG imaging and RSM imaging, CESM can show the mass and shape of the tumor, as well as the characteristics of malignant calcification and enhancement. In clinical practice, breast cancer patients showed similar enhancement in CESM and CE-MRI, and the morphological descriptors for these two techniques were also similar [22]. CE-MRI contributed to the MMBC diagnosis based on the shape and enhancement curve of the tumor and the signal characteristics of DWI; however, its specificity was comparatively low in a range of 37%–97% [23], as it could not show the characteristic calcification of breast malignancy. This would result in invasive diagnostic tests (e.g., core needle biopsy) that were not necessary. Some scholars concluded that CESM was superior to MRI in detecting noninvasive carcinomas, especially if there were only clustered calcifications in the lesions. Previous studies showed that the specificity of CESM was up to 90% [11]. Our results also confirmed that the specificity of CESM was higher than that of CE-MRI (36.4% vs 63.6%). Among the 177 malignant, 54 lesions (30.51%) showed clustered microcalcifications in the LE-MG imaging. Thirty-five lesions (64.8%) were assessed as BI-RADS 5, while for CE-MRI, 22 (40.7%) were diagnosed as BI-RADS 5. Therefore, CESM LE-MG imaging can detect more malignant calcifications in the breast than CE-MRI, which increased the confidence in the diagnosis of breast cancer.

CESM showed different enhancement in RSM imaging between benign and malignant lesions. Benign lesions showed weak or no enhancement. Among the 165 malignant lesions detected by CESM, 160 (96.9%) lesions were IDC, in which 154 (96.3%) lesions presented markedly heterogeneous enhancement and the other 6 lesions (3.7%) showed mild enhancement. All the 5 DCIS were manifested as mild enhancement. Hence, IDC was mainly manifested as severe heterogeneous enhancement, while DCIS was mainly manifested as mild enhancement. IDC lesions presented higher enhancement than that of DCIS. Our data also showed that non-mass lesions with mild enhancements or clustered microcalcification lesions with mild enhancements were closely related to DCIS (100%, 5/5), which was concordant with that of the previous literature description [24]. This was speculated to be associated with more aggressive behavior and abundant blood flow of IDC than DCIS. In a previous study, approximately 11% of the high-grade DCIS showed no enhancement [25]. In our study, none of the patients showed such type of breast cancer, which may be related to the fact that the sample size for the carcinoma in situ was relatively small. Interestingly, the smallest DCIS in the CESM images showed a diameter of 3 mm. In our future study, we will focus on finding more characteristics of breast cancer to improve the diagnostic confidence of CESM.

In addition, CESM could provide a more intuitive image, which was beneficial to the preoperative localization of lesions. We found a special case occasionally. In the CESM images of the patients, there was a malignant mass and a nodule (about 3 mm in diameter) with significant enhancement in the subcutaneous tissues of the nipple. The morphology and location were consistent on both CESM and CE-MRI. A small hemangioma was confirmed after surgery (Figure 4). Obviously, it was easier and more convenient to find out the small nodules based on CESM images. In addition, the body position for CE-MRI was prone position not the supine position. Therefore, the localization of small nodules in breast was more difficult in CE-MRI than that of CESM.

There are some limitations for CESM. For example, it required close cooperation of the patients. During the CESM scan, the breast cancers in the inner quadrant of the breast adjacent to the chest wall were more likely to be neglected. One patient with tumor in the deep internal quadrant close to the chest wall was misdiagnosed as she felt pain after puncture at the wound site (Figure 5). Therefore, CESM examination must be performed prior to targeted puncture. In addition, in order to maximally include all the breast tissues, muscle relax in the thoracic wall was recommended.

Eleven benign lesions were misdiagnosed as MMBC including 5 lesions of fibroadenoma, 3 lesions of fibrocystic lesion with ductal hyperplasia, 2 lesions of breast adenosis with fibroadenoma, and 1 lesion of ductal dilatation of the breast. Seven lesions were misdiagnosed as MMBC by CE-MRI, and four lesions were misdiagnosed as MMBC by CESM. Breast adenosis, fibroadenoma, and ductal dilatation of the breast cases were all presented multifocal and mild enhancement due to which it was difficult to distinguish DCIS. This is associated with the small sample size for carcinoma in situ, together with a lack of experience on the differential diagnosis. This is a retrospective analysis. All the cases included in this study received CESM and MRI within 3–14 days. In our hospital, we can only perform US-guided puncture, rather than X-ray-guided or MRI-guided puncture. In cases of few small lesions or multiclustered calcification by X-ray or by MRI, which cannot be detected by US, it is still difficult to remove lesions surgically.

Compared with MR diagnosis, CESM showed the characteristics of less time-consuming, low cost, and sensitivity to calcification; however, it was still a challenge to wrap all of the mass adjacent to the chest wall as it may result in FN. MRI had the advantages of being able to image the entire chest wall and axilla, and it involved no ionizing radiation. Although iodinated contrast was generally considered to be significantly more hazardous than gadolinium contrast, whether the deposition of gadolinium had any actual consequences to human health was unknown.

## 5. Conclusions

In conclusion, CESM can display breast lesions and has diagnostic efficacy equivalent to CE-MRI in detecting MMBC. CESM promoted the identification of MMBC, which was beneficial to the surgery selection, generation of negative surgical margins, and avoiding treatment failure.

## Figures and Tables

**Figure 1:** Imaging features of a 54-year-old female with left-sided MMBC. (a) Breast US indicated only an irregular solid hypoechoic mass in the left breast (triangle), which was diagnosed as BI-RADS 4C. (b) MLO position in left breast. In CESM, the LE-MG imaging indicated two masses with unclear and irregular edges in the outer upper quadrant of the breast (arrow). (c) In CESM, the RSM imaging indicated the weak and significantly heterogeneous enhancement of masses. Two masses were diagnosed as BI-RADS 4C. (d, e) The patient received CE-MRI again due to disputes in the results of the US and CESM. The MIP imaging obtained after CE-MRI at transverse and coronal views. They indicated two significantly heterogeneous enhancements of masses with spiculated edges (arrows), which were diagnosed as BI-RADS 4C. (f) The posterior mass was confirmed to be invasive lobular carcinoma after surgery. The HE staining results were observed under a magnification of 10×. (g) The anterior mass was invasive lobular carcinoma and DCIS. HE staining results were observed under a magnification of 20×.

**Figure 2:** Imaging features of a 39-year-old woman with MMBC in the right breast. (a) CC position in the right breast. In CESM, the LE-MG imaging indicated a star-shaped mass in the outer quadrant of the right breast (arrow). (b) In CESM, the RSM imaging indicated six slightly enhanced masses with irregular edges and not circumscribed margin (arrows). (c) Enlarged LE-MG imaging: there were clusters of fine linear branching calcifications. Combined with the RSM imaging, the six small masses were diagnosed as BI-RADS 5. (d) US indicated only two hypoechoic masses with irregular edges (crosses), which was classified as BI-RADS 4A. Six masses were confirmed as IDC after surgery. (e) The pathology features of HE under a magnification of 20×. (f) The smallest mass was DCIS with a diameter of 3 mm. The HE staining results were observed under a magnification of 10×.

**Figure 3:** Imaging features of a 45-year-old woman with MMBC in the left breast. (a) CC position in the left breast. In CESM, the LE-MG imaging indicated dense breast parenchyma with no suspicious findings. (b) In CESM, the RSM imaging indicated the first mass with irregular edge and significantly heterogeneous enhancement in the outer quadrant (arrow), which was diagnosed as BI-RADS 4C. The second and third irregular masses along the duct were seen in the inner quadrant, with mild enhancement (triangles). They were diagnosed as BI-RADS 4B. (c) US indicated a hypoechoic nodule with irregular edge (triangles), which was diagnosed as BI-RADS 4C. (d–f) T1WI image of CE-MRI fat compression in axial position showed three nodules in the left breast. The morphology and location were consistent both on CESM and CE-MRI. They were also diagnosed as BI-RADS 4C and 4B, respectively (arrows). (g) The first mass was confirmed to be IDC after surgery by HE staining under a magnification of 20×. (h) The second and third masses were DCIS, by HE staining under a magnification of 10×.

**Figure 4:** Imaging features of a 45-year-old woman with breast cancer in the right breast. (a) MLO position in the right breast. In CESM, the LE-MG imaging indicated dense breast parenchyma with no suspicious findings. (b) In CESM, the RSM imaging indicated the first mass with long spiculated edge, with significantly heterogeneous enhancement (wide arrow), which was diagnosed as BI-RADS 5. Under the right papilla, there was another small mass with significant enhancement and round margin (narrow arrow), which was diagnosed as BI-RADS 3. (c, d) T1WI image of CE-MRI fat compression in axial position: the morphology and location of the two lesions were consistent on both CESM and CE-MRI, which were diagnosed as BI-RADS 5 and 3, respectively. (e) US indicated only a hypoechoic mass with irregular edge (crosses), which was diagnosed as BI-RADS 4C. (f) It was confirmed that the first mass was an IDC, as revealed by HE staining under a magnification of 20×. The second mass was a small subcutaneous hemangioma.

**Figure 5:** Imaging features of a 50-year-old woman with MMBC in the right breast. (a, b) CC position in the right breast. In CESM, the LE-MG and RSM imaging indicated asymmetric density shadow in the inner quadrant, with mild ductal enhancement (wide arrow). (c, d) MLO position in the right breast. In CESM, the LE-MG and RSM imaging indicated asymmetric density shadow in the lower quadrant, with mild ductal enhancement (wide arrow). The diagnosis was BI-RADS 4A. The pectoralis major muscle was not well displayed, which may not be diagnosed. (e) US indicated a hypoechoic mass with irregular edge (crosses), which was diagnosed as BI-RADS 4C. (f, g) T1WI image of CE-MRI fat compression in axial position showed the first mass with irregular and heterogeneous enhancement, which could be seen in the lower inner quadrant of the right breast (wide arrow). The second lesion showed non-mass and ductal enhancement around the mass (wide arrow). (h) The first mass was confirmed to be IDC after surgery, as shown in HE staining under a magnification of 20×. (i) The non-mass lesion was DCIS, as shown in HE staining under a magnification of 10×.

**Table 1:** Number of suspicious lesions of CESM and CE-MRI in detecting MMBC.

Viable	Number of suspicious lesions	True-positive value	False-positive value	False-negative value	True-negative value
CESM	178	174	4	3	7
CE-MRI	183	176	7	1	4

**Table 2:** Comparison between the diagnostic efficacy of CESM and CE-MRI in detecting MMBC.

Variable	CESM	CE-MRI	CESM vs. CE-MRI	
			*p* value	*χ* ^2^
Sensitivity	98.3% (174/177)	99.4% (176/177)	0.500	0.500
Specificity	63.6% (7/11)	36.4% (4/11)	0.250	1.333
Accuracy	96.3% (181/188)	95.7% (180/188)	0.792	0.069

## Data Availability

The data that support the findings of this study are available from the corresponding author, upon reasonable request.
